This article has been retracted.

# Relay cropping of cotton in wheat improves productivity of cotton-wheat cropping system

**DOI:** 10.1371/journal.pone.0266694

**Published:** 2022-04-14

**Authors:** Muhammad Tariq, Muhammad Naveed Afzal, Muhammad Ahmad, Zeeshan Ahmed, Muhammad Umer Afzal, Amir Maqbool, Abdulrahman Al-Hashimi, Mohamed S. Elshikh

**Affiliations:** 1 Agronomy Section, Central Cotton Research Institute, Multan, Pakistan; 2 Xinjiang Institute of Ecology and Geography, Chinese Academy of Sciences, Urumqi, Xinjiang, China; 3 CIMMYT International, Pakistan Office, Islamabad, Pakistan; 4 Institute for Integrative Biology of the Cell (I2BC), Université Paris-Saclay, CNRS, Gif-sur-Yvette, France; 5 Department of Botany and Microbiology, College of Science, King Saud University, Riyadh, Saudi Arabia; Ghazi University, PAKISTAN

## Abstract

Cotton-wheat (CW) is an important cropping system in Pakistan; however, delayed cultivation of cotton after wheat significantly deceases system productivity. Late-sown cotton crop suffers from heat stress, high fruit shedding and infestation of various pests and cotton leaf curl virus (CLCV). Therefore, early sowing of cotton is preferred to overcome these challenges. However, cotton planting is overlapped with the harvesting of wheat crop in CW cropping system. Since fallow land is unavailable, relay intercropping of cotton in wheat crop seems a viable option for early planting. This three-year field study evaluated the role of relay cropping of cotton in improving the productivity of CW cropping system and lowering CLCV infestation. Wheat was planted in 22.5 cm rows with no row skipped (W_1_), one row skipped after every three (W_2_), and six rows (W_3_) for planting cotton in 0.75 and 1.50 m apart rows. Early cotton was planted in fallow land (C_1_) and standing wheat in 0.75 (C_2_) and 1.50 m (C_3_) apart rows and conventional planting after wheat harvesting (C_4_). Yield losses of wheat crop ranged from 8.16 to 19.81% in W_3_ and W_2_, respectively compared W_1_. However, C_2_ and C_3_ treatments improved cotton yield by 86.07% and 64.89% suppressed CLCV infestation by 68.14% and 65.86%, respectively compared to C_4_. Moreover, net benefits from relay cropping (W_2_C_2_) were 2190.1 $ ha^-1^ in 2013–14, 1954.4 $ ha^-1^ in 2014–15 and 2559.5 $ ha^-1^ in 2015–16 in comparison with C_1_ (1543.5, 1311.7 and 1892.3 $ ha^-1^ during 2013–14, 2014–15 and 2015–16, respectively). The W_2_ resulted in higher cotton yield compared to W_3_ which is mainly attributed to double number of cotton rows in W_2_ than W_3_. It is concluded that cotton relay cropping (W_2_C_2_) resulted in the highest economic returns with minimum CLCV infestation. Therefore, W_2_C_2_ is recommended for improving the system productivity of CW cropping system.

## Introduction

Cotton-wheat (CW) is the second most important cropping systems in South Asia after wheat-rice spanning over an area of ~4.19 mha in India and Pakistan [1]. The system provides cotton fiber, and wheat grains for food security and farmer’s income. Generally, cotton cultivation is followed by wheat in CW system, and no fallow period is the most important issue of this system. The sowing of succeeding crop gets late because of overlapping harvesting period of preceding crop [2–6]. Late-sown cotton crop faces multiple stresses during different growth and developmental stages. The targeted cotton yield is not being achieved in Pakistan since the last two decades due to various biotic and abiotic constraints and all of which are responsible for delayed planting of cotton crop [7–9].

Generally, cotton is sown during mid-April and picked/harvested in October. However, late sowing results in impair seed germination, root shoot ratio, and seedling establishment due to high temperature [10, 11]. Likewise, late planting pushes peak boll development period to cold weather which results in lower number of opened bolls. Although different agronomic approaches such as seed priming, mixed cropping or crop rotation have been employed to improve seed germination and production of cotton crop in CW cropping system, yield remains low. Several studies have demonstrated potential yield benefits for early planting in cotton crop [4, 8, 9, 12]. Cotton leaf curl virus (CLCV) in Pakistan was initially reported in 1967 and its severity remained mild until 1990s. It drastically reduced total cotton production from 12.82 to 9.82 million bales within two years from 1991–92 to 1993–94 [13–15].

Several management and genetic improvement approaches have been employed since 1994 for reducing CLCV infestation in Pakistan. The peak CLCV infestation is recorded during 27^th^ to 31^st^ week of the year, regardless of the sowing time and genotypes [16]. Early planting enables cotton to complete its growth and boll setting during disease-free period. Meanwhile, late planted crop faces CLCV infestation at early growth stages, resulting in stunted growth. Several studies have concluded that early planting is a better choice for escaping CLCV infestation [9, 17, 18]. Furthermore, prolonged growth season and low CLCV infestation are the main contributor towards higher yield of early planted cotton [8, 9, 18]. Although development and cultivation of transgenic cotton (Bt-cotton) assisted in improving cotton production in Pakistan, it could not fulfill the demands of the country [14].

Besides high yield and disease escape, early planting got popular with the introduction of Bt-cotton in the country during early 2000s. It was due to inherent resistance against certain insects and improved boll setting ability of Bt-cotton over entire growth season [4, 19]. Higher yield benefits, low disease infestation and better economic returns forced the farmers to keep land fallow during winter for spring planting of cotton. It was likely to reduce the wheat cultivation area in future and considered as a potential threat for national food security since >50% wheat comes from CW cropping system [4, 20].

Relay cropping is one of the practical approaches to resolve the time conflict (3–4 weeks) between wheat harvesting and cotton sowing in CW cropping system [2, 4, 21]. Relay cropping is an intercropping system in which second crop is sown on onset of reproductive growth of first crop so that a full space is available after the harvest of the first crop [4, 5, 21]. It intensifies the system through time, and recommended method for areas characterized with short growing season [22]. The most important advantages of relay cropping are higher yield with efficient use of available resources from the same piece of land in a specific time [5]. The basic objective of relay cropping is to extend the growing season of second crop by early planting. However, it is important to develop strategy for minimizing the damage to first crop during sowing and to second crop while harvesting first crop [23]. Potential benefits of relay intercropping of wheat-potato [24], rice-chickpea [25], red clover-wheat [26], legumes-millet [27], legumes-maize [28], lentil-rice [29] and muskmelon-strawberry [30] have been previously documented.

Initially, relay cropping in cotton-wheat cropping system was implemented by broadcasting wheat seed in standing cotton crop [2, 3, 6, 31]. Since early 2000s, the feasibility of various techniques to plant cotton in standing wheat is being investigated in China and Pakistan [4, 20, 32–34]. The techniques used so for are labor-intensive and unconducive to mechanization. Moreover, potential of relay cropping as management strategy for CLCV in CW cropping system and its efficiency have not been investigated yet. We hypothesize that relay cropping of cotton in skipped wheat rows may improve economic returns and lower CLCV infestation. To do this, some modifications in wheat sowing pattern such as managing row spacing and skipping rows are required for successful planting. In Pakistan, wheat is drilled at 22.5 cm apart rows and cotton is planted in 0.75 m apart rows. Therefore, wheat row can be skipped at specified distance to make cotton planting convenient. The experiment was designed by skipping the cultivation of wheat in few rows during winter season and cotton was relay planted in skipped rows during summer season to overcome problems associated with delayed sowing. The main objectives of the study were to lower CLCV disease through early planting, use of minimum tillage and improving profitability CW cropping system.

## Materials and methods

### Soil and weather

Three years (2013–16) field study was conducted at agronomic research area of Central Cotton Research Institute (CCRI), Multan, Pakistan (30°12’N, longitude 71°28’E and altitude 123 m a.s.l). The soil of the experimental site was alkaline (pH = 8.1), poor in organic matter (1.1%) and silt-loam in texture with good drainage. The metrological data were recorded by weather station in the vicinity (300 m) of experimental site. The climate of experimental area was arid due to high evaporation rate, mean maximum (30.01°C) and minimum daily temperature (19.96°C). The daily mean relative humidity and total average annual rainfall was 71.64% and 255.26 mm, respectively (Table 1).

**Table 1:** Metrological conditions of experimental area.

Months	Av. max. temperature (˚C)	Av. min. temperature (˚C)	Mean relative humidity (%)	Total rainfall (mm)
November 2013	26.9	13.1	79.1	0.0
December 2013	20.4	9.3	50.4	0.0
January 2014	19.7	6.2	55.3	1.5
February 2014	21.2	8.6	81.8	18.0
March 2014	25.4	14.2	74.2	33.4
April 2014	33.6	20.2	55.1	8.9
May 2014	36.7	24.6	53.9	42.6
June 2014	39.9	30.5	52.3	1.4
July 2014	36.8	29.4	61.1	51.6
August 2014	35.7	28.4	71.2	16.5
September 2014	34.1	25.6	75.5	4.3
October 2014	31.5	20.5	73.2	17.7
November 2014	26.3	12.0	77.0	0.0
December 2014	17.8	6.9	84.3	0.0
January 2015	17.7	6.7	88.0	0.8
February 2015	21.7	10.9	74.9	4.0
March 2015	25.2	15.3	73.3	92.9
April 2015	34.7	22.2	65.4	9.2
May 2015	38.7	26.4	53.1	8.5
June 2015	37.7	28.9	56.2	24.5
July 2015	34.5	28.2	71.5	151.2
August 2015	33.9	31.1	77.6	67.0
September 2015	33.8	28.0	85.2	15.4
October 2015	31.3	22.0	73.5	7.0
November 2015	25.1	14.9	65.0	0.0
December 2015	20.6	9.7	75.1	0.0
January 2016	16.4	9.9	85.9	0.9
February 2016	23.2	10.7	74.6	0.1
March 2016	26.1	17.8	77.5	20.1
April 2016	34.5	22.5	86.0	13.1
May 2016	40.2	28.5	74.3	2.0
June 2016	39.8	31.1	69.1	4.0
July 2016	36.5	29.5	73.0	36.2
August 2016	35.1	28.1	84.6	109.0
September 2016	34.8	26.2	82.7	4.0
October 2016	33.0	20.8	68.9	0.0

### Wheat crop husbandry

Wheat seeds were drilled in 22.5 cm spaced rows by using 120 kg seed per hectare on 28^th^ November, 8^th^ December and 28^th^ December in 2013, 2014 and 2015, respectively. The treatments were conventional wheat sowing at 22.5 cm space (W_1_), every 4^th^ (W_2_) and 7^th^ wheat row skipped (W_3_) for making cotton planting convenient in standing wheat. Wheat crop was fertilized with 125 kg N ha^-1^ in three splits (pre-sowing, first irrigation and booting stage) and 100 kg P_2_O_5_ ha^-1^ as pre-sown application. The 4^th^ and 7^th^ row was skipped for cotton planting in 0.75 and 1.50 m apart rows, respectively. This made 22.5 cm space available for cotton planting between rows, while space occupied by wheat was used as tractor track and implements after wheat harvesting. A 1 m^2^ area was manually harvested at maturity during end of April to record grain yield of wheat crop.

### Cotton crop husbandry

The transgenic cotton cultivar (‘CIM-616’) was planted as monoculture on fallow land for C_1_, in standing wheat at 0.75 m (C_2_) and 1.50 m distance (C_3_) and conventional planting after wheat harvesting (C_4_). It resulted in a ratio of one row of cotton in three (1:3) and six (1:6) rows of wheat in C_2_ and C_3_, respectively (Fig 1).

**Fig 1:** Layout of various relay cropping treatments used in the current study.

Light irrigation was applied to wheat field before cotton sowing as relay crop (C_2_ and C_3_). The cotton in standing wheat was planted during 4^th^ & 8^th^ April in 2014 and 2015, and 18^th^ March in 2016. Cotton in C_1_ was planted on 5^th^ April, 8^th^ April and 19^th^ April during 2014, 2015 and 2016, respectively. The conventional planting (C_4_) was done on 30^th^ May, 04^th^ June and 20^th^ May during 2014, 2015 and 2016, respectively. The system is divided in three phases i.e., wheat phase, wheat-cotton intercrop, and cotton phase. The crop was fertilized with 150 kg N ha^-1^ from urea by fertigation methods in four equal splits. The wheat and cotton shared about 5 weeks of overlapped growth period where reproductive development of wheat was overlapped with seedlings stage of cotton. The seed cotton yield was recorded by manual picking of fully opened bolls. Data on bolls (m^-2^) and boll weight were recorded from three randomly selected places and hundred opened bolls, respectively. The CLCV incidence was recorded periodically at 15-days interval from 1^st^ June to 30^th^ September and presented as incidence (%).

### Economic and statistical analysis

The land use, production efficiency and profitability were calculated. Land use efficiency was calculated by dividing the number of cropping days to the total number of days in a year. The production efficiency was determined by dividing total production of cropping system to the total number of days of a year. The formula for land use and production efficiency are given below [35] [36]

$$Land\;use\;efficiency\;(\%)=\frac{D1+D2\;}{365}\times 100$$

The D1 and D2 are number of cropping days of first and second crop in a cropping system

$$Production\;efficiency\;(\%)=\frac{Y1+Y2}{D1+D2}\times 100$$

The Y1 and D1 are yield and duration first crop, while Y2 and D2 are yield and duration of second crop, respectively.

The profitability (income per day) was worked out by following the procedure of Mukherjee [37].


$$Profitability\;(US\$\;{day}^{-1}\;{ha}^{-1})=\frac{Total\;net\;income\;of\;cropping\;system}{Total\;cropping\;duration}$$

The economic analysis was carried to determine the profitability of cotton wheat relay cropping including all the expenses from sowing to harvesting of both crops. Benefit cost ratio (BCR) was estimated using prevailing average cost of inputs and value of produce. Statistix 8.1 software was used for analysis of variance and means comparison was carried out through least significant difference test (LSD) at 5% probability level [38].

## Results

### Yield and related traits of wheat and cotton

The results indicated that number of productive tillers and grain yield of wheat were significantly affected by different planting treatments, whereas number of grains per spike and 1000-grain weight remained unaffected (Fig 2). The highest number of productive tillers were recorded in W_1_ followed by W_3_ and W_2_. Wheat sown in W_2_ and W_3_ produced 19.5 and 9.2% lesser grain yield than W_1_ during 2014. Significant reduction in number of productive tillers was observed in 2015. The tillers were reduced by 19.9% and 9.5% in W_2_ and W_3_ compared to W_1_. Meanwhile, grain yield was decreased by 20.3% in W_2_ and 8.9% in W_3_ during 2015 in comparison with W_1_. The number of productive tillers and grain yield were reduced by 23.2 and 11.4%, and 19.6 and 6.4%, respectively during 2016.

**Fig 2:** Grain yield and yield components of wheat sown in under different planting techniques. In X-axis legend, W_1_ = conventional wheat sowing in 22.5 cm spaced rows, W_2_ = every 4^th^ wheat row skipped and W_3_ = every 7^th^ wheat row skipped for relay cropping of cotton in wheat.

There were significant variations among planting treatments for plant height, number of bolls and seed cotton yield (Fig 3). Similar plant height was noted for cotton sown in C_1_, C_2_ and C_3_ during 2014; however, it was higher than C_4_. Relayed cropped cotton in C_2_ produced similar number of bolls (m^-2^) and seed cotton yield with C_1_. Cotton sowing in C_4_ resulted in the lowest number of bolls and seed cotton yield. Plant height, bolls, and seed cotton yield in C_4_ were statistically lower than rest of the treatments. However, C_1_, C_2_ and C_3_ were non-significant with each other for plant height. The C_1_ and C_2_ produced statistically similar number of bolls and seed cotton, which were higher than C_4_ and C_3_. The similar results as of 2014 were recorded during 2015 and 2016. The yield was improved by 89.7%, 89.6% and 68.7% in C_1_, C_2_ and C_3_, respectively over C_1_ during 2016. The results of three years experimentation showed that relay cropped cotton in C_2_ produced equal yield with C_1_ indicating that C_2_ can be adopted as an alternative to C_1_.

**Fig 3:** Plant height, seed cotton yield and related traits of cotton sown under different planting techniques. In X-axis legend, C_1_ = cotton grown as sole crop, C_2_ = relay cropped cotton in wheat (75 cm apart rows), C_3_ = relay cropped cotton in wheat (150 cm apart rows) and C_4_ = cotton planting after wheat harvesting.

The CLCV infestation was significantly influenced by different planting techniques used in the study. The differences in CLCV infestation during 2014 were non-significant in C_1_, C_2_, C_3_; however, these treatments observed low CLCV infestation compared to C_4_. Similar trend was observed during 2015. Moreover, relay cropped cotton (C_2_ and C_3_) observed the lowest CLCV infestation during 2016. The highest CLCV infestation during 2016 was noted for C_4_ (Fig 4).

**Fig 4:** Cotton leaf curl virus incidence on cotton crop sown under various planting techniques. In X-axis legend, C_1_ = cotton grown as sole crop, C_2_ = relay cropped cotton in wheat (75 cm apart rows), C_3_ = relay cropped cotton in wheat (150 cm apart rows) and C_4_ = cotton planting after wheat harvesting.

### Economic performance of relay cropping

The economic analysis revealed that costs incurred on wheat cultivation in W_1_, W_2_ and W_3_ ranged between 487.1 and 507.5, 522.7 and 543.8 and 516.0 to 540.2 $ ha^-1^ during 2013–14, 2014–15 and 2015–16, respectively. The income generated from these treatments varied between 1127.9 to 1404.2, 1158.0 to 1457.9 and 1162.1 to 1355.6 $ ha^-1^ during 2013–14, 2014–15 and 2015–16, respectively. The minor differences in production costs resulted in 3 to 5 times higher income of wheat crop. Regarding cotton, the differences in cultivation cost differed from 1070.7 to 1384.3, 1091.2 to 1427.9 and 1048.0 to 1444.4 $ ha^-1^ during 2013–14, 2014–15 and 2015–16, respectively. The income ranged from 1537.3 to 2917.1, 1433.6 to 2739.6 and 1755.0 to 3330.1 $ ha^-1^ during 2013–14, 2014–15 and 2015–16, respectively. Although the seasonal net benefits of cotton remained the highest when crop was sown on fallow land, results were inconsistent at cropping system level. The highest net returns of 2190.1, 1954.4 and 2559.5 $ ha^-1^ during 2013–14, 2014–15 and 2015–16 were noted for relay cropped cotton in 0.75 m rows (W_2_C_2_). It was closely followed by treatment in which cotton was sown alone on fallow land (Table 2).

**Table 2:** Economic analysis of cotton and wheat production in different cotton-wheat relay planting systems.

Wheat					Cotton				Cropping system profitability			
**Treatments**	**Fixed cost** ($ ha^-1^)	**Variable cost** ($ ha^-1^)	**Expense** ($ ha^-1^)	**Income** ($ ha^-1^)	**Fixed cost** ($ ha^-1^)	**Variable cost** ($ ha^-1^)	**Expense** ($ ha^-1^)	**Income** ($ ha^-1^)	**Total expenses** ($ ha^-1^)	**Gross income** ($ ha^-1^)	**Net profit** ($ ha^-1^)	**Benefit cost ratio**
**2013–14**												
W_1_C_4_	425.9	81.6	507.5	1404.2	120.8	949.9	1070.7	1537.3	1578.2	2941.5	1363.3	1.86
W_2_C_2_	425.9	61.2	487.1	1127.9	120.8	1244.3	1365.0	2914.3	1852.1	4042.2	2190.1	2.18
W_3_C_3_	425.9	69.9	495.8	1275.3	120.8	1263.5	1384.3	2594.0	1880.1	3869.3	1989.2	2.06
C_1_	-	-	-	-	120.8	1252.8	1373.6	2917.1	1373.6	2917.1	1543.5	2.12
**2014–15**												
W_1_C_4_	458.2	85.6	543.8	1457.9	122.3	968.9	1091.2	1433.6	1635.0	2891.5	1256.5	1.77
W_2_C_2_	458.4	64.2	522.7	1158.0	122.3	1260.7	1383.0	2702.1	1905.7	3860.1	1954.4	2.03
W_3_C_3_	458.4	73.4	531.8	1328.1	122.3	1288.2	1410.5	2403.3	1942.3	3731.4	1789.1	1.92
C_1_	-	-	-	-	122.3	1305.6	1427.9	2739.6	1427.9	2739.6	1311.7	1.92
**2015–16**												
W_1_C_4_	445.3	94.9	540.2	1448.1	93.3	954.7	1048.0	1755.0	1588.2	3203.1	1614.9	2.02
W_2_C_2_	444.9	71.2	516.0	1162.1	93.3	1320.3	1413.6	3327.0	1929.6	4489.1	2559.5	2.33
W_3_C_3_	444.9	81.3	526.2	1355.6	93.3	1351.1	1444.4	2961.4	1970.6	4317.0	2346.4	2.19
C_1_	-	-	-	-	93.3	1344.5	1437.8	3330.1	1437.8	3330.1	1892.3	2.32

W_1_C_4_ = conventional wheat-cotton sowing, W_2_C_2_ = wheat-cotton relay cropping system (R×R = 75 cm), W_3_C_3_ = wheat-cotton relay cropping system (R×R = 150 cm), C_1_ = cotton as sole crop (R×R = 150 cm),—indicates that computation was not possible.

The data further revealed that loss wheat grain yield loss in W_2_ and W_3_ for cotton relay cropping should not be considered as a significant economic loss since it can be compensated from higher seed cotton yield which has two times high unit price than wheat. The performance of various planting treatments was in term of economics, land use and production efficiency are given in Table 3. The total cropping duration and system productivity differed across various treatments. The highest duration, land use and production efficiency were recorded for relay cropping treatments W_2_C_2_ and W_3_C_3_, whereas monocrop cotton resulted in the lowest values for these parameters. Cotton monocrop (C_4_) recorded higher values for daily profitability because it is only for cotton season (about 8 month) rather than whole year as for other treatments.

**Table 3:** System productivity, land use and profitability of wheat-cotton relay cropping techniques used in the current study.

Treatments	Wheat duration (days)	Cotton duration (days)	Total duration of cropping system (days)	System productivity (kg ha^-1^)	Land use efficiency (%)	Production Efficiency (kg ha^-1^ day^-1^)	Profitability ($ ha^-1^ day^-1^)
2013–14							
W_1_C_4_	166	172	338	7086.6	92.6	19.4	4.03
W_2_C_2_	166	228	394	8256.3	107.9	22.6	5.56
W_3_C_3_	166	228	394	8169.6	107.9	22.4	5.05
W_1_C_4_		227	227	4588.1	62.2	12.6	6.80
2014–15							
W_1_C_4_	163	192	355	6903.5	97.3	18.9	3.54
W_2_C_2_	163	249	412	7989.7	112.9	21.9	4.74
W_3_C_3_	163	249	412	8040.7	112.9	22.0	4.34
W_1_C_4_		249	249	4372.8	68.2	12.0	5.27
2015–16							
W_1_C_4_	124	199	323	6833.2	88.5	18.7	5.00
W_2_C_2_	124	262	386	8145.1	105.8	22.3	6.63
W_3_C_3_	124	262	386	8220.4	105.8	22.5	6.08
W_1_C_4_		261	261	4606.7	71.5	12.6	7.25

W_1_C_4_ = conventional wheat-cotton sowing, W_2_C_2_ = wheat-cotton relay cropping system (R×R = 75 cm), W_3_C_3_ = wheat-cotton relay cropping system (R×R = 150 cm), C_1_ = cotton as sole crop (R×R = 150 cm).

## Discussion

Different planting techniques exerted significant impacts on crop yields and productivity of CW cropping system in the current study. Wheat sowing according to W_2_ and W_3_ produced less grain yield than W_1_ since a significant portion of land was left unseeded due to skipped rows for cotton planting between rows. It reduced overall plant population, density of productive tillers and grain yield. However, yield loss was comparatively less in W_3_ than W_2_ due to higher plant population. Despite 25 and 14% reduction in number of wheat rows in W_2_ and W_3_, the corresponding yield reductions was 20.3 and 9.2%, respectively. Relatively low yield reduction in comparison with reduction is number of rows is due to higher tillering in outer rows. It compensates the yield losses to some extent. It has been reported in literature that yield of companion crop is decreased in intercropping due to strong competition for natural resources [39]. However, the yield reduction in the current study was mainly due to low plant population because of skipped wheat rows. Low wheat grain yield in relay cotton and maize has been witnessed in earlier studies [4, 40]. Relative low grain yield was recorded during 2016 because of late sowing and prevalence of relatively high temperature during March (Table 1) which impaired normal development of grains.

Cotton planting in wider rows availed equal growth period; however, produced lower yield due to sub-optimal plant population. Although C_3_ had half number of rows compared to C_2_, reduction in number of bolls and seed cotton yield was only 13.4 and 12.3%, respectively. The plants from outer rows availed more space and produced long branches to compensate yield losses caused by a smaller number of rows. Significant yield differences can be linked with the extra two months growth period resulting from early planting. Crop sown during the end of March or early April attained significant height before the onset of heat stress during June and July (Table 1) and CLCV incidence which is quite clear from Fig 4. Irrespective of crop age, CLCV incidence is favored by small differences in day and night temperature. Such conditions are naturally available from mid-July to end of August (Table 1). The early planted cotton had sufficient CLCV-free growth period and better tolerated its infestation in the current study. Previous studies also reported low CLCV infestation on early sown crop [9, 18].

Yield of relay cropped cotton (C_2_ and C_3_) ranged from 3992.9 to 4505.7 kg ha^-1^ corresponding to 0.37 and 11.71% decrease compared to C_1_. On the other hand, C_2_ and C_3_ produced 86.07 and 64.9%, more seed cotton yield, respectively compared to C_4_. Higher seed cotton yield in fallow land and relay cropping treatments due to prolonged growth period to produce more bolls and sufficient time for boll opening. Overall cotton performance in 2015 was poor due to excessive rainfall (Table 1).

Higher seed cotton yield in cotton relay cropping is in line with earlier studies [4, 19, 41, 42]. In contrast to our results, the lower seed cotton yield has been reported over sole crop in China due to poor light availability [33]. However, light availability was not an issue in the current study and standing wheat provided protection to young cotton plants from hot wind. Therefore, yield of relay system was not less than fallow land planting (Fig 3). Relay cropping of cotton although produced statistically similar yield, but the technique also permits the cultivation of wheat which is an additional benefit in contrast to sole cotton sowing.

Economic analysis is important for the social acceptance of relay cropping among the farmers [43–45]. Better economics returns, land use and production efficiency of cotton relay cropping was due to timely planting and low production costs, mainly invested in conventional seedbed preparation [4]. The cost of cultivation for wheat varied for sowing, irrigation, weeding, plant protection and picking (Table 3). Although cotton planting after wheat harvesting had less economic benefit over cotton planting as sole, exclusion of wheat is not a good decision national food security. Data in Table 2 revealed better economic return of cotton-wheat cropping system were based on existence of cotton either its sole cultivation or relay cropped with wheat. The higher cotton yield in relay cropping also compensate the economic losses of low yield from skipped wheat rows for cotton sowing as relay. The decision of producing only cotton is good if higher market prices exist. The unit price of cotton varies greatly from year to year and decision of cotton planting after wheat or fallow land depends on the cotton prices. Considering the greater flexibility in cotton prices and wheat role in national food security, it is recommended that exclusion of wheat from system should not be compromised, where relay cropping is potential tool for ensuring higher profitability and food security [20].

## Conclusions

Skipped rows planting system of wheat decreased its yield; however, resulted in higher yield of cotton. It was observed that relay planting did not reduce the cost of cultivation but likely to improve the productivity of cropping system. Although, skipped rows in wheat produced less yield but maintained the higher returns round the year through higher cotton yield. Furthermore, relay cotton planting in late March is a better choice to manage cotton leaf curl virus infestation and increase system productivity by extending the growing season rather to exclude wheat by keeping land fallow for early planting of cotton. It ensures good economic returns and higher system productivity in comparison to conventional planting system after wheat harvesting which is characterized with low yield due to high cotton leaf curl virus attack.

## References

[1] SinghY, KukalSS, MangiLJ, HarminderSS. Improving water productivity of wheat-based cropping systems in South Asia for sustained productivity. Adv Agron. 2014; 127: 157–258.

[2] KhanMB, KhaliqA. Production of winter cereals as relay crops by surface seeding in cotton-based cropping system. J Res (Sci). 2005; 16: 79–86.

[3] ButtarGS, SidhuHS, SinghV, JatML, GuptaR, SinghY, et al. Relay planting of wheat in cotton: an innovative technology for enhancing productivity and profitability of wheat in cotton–wheat production system of South Asia. Exp Agric. 2013; 49: 19–30.

[4] ShahMA, FarooqM, HussainM. Productivity and profitability of cotton–wheat system as influenced by relay intercropping of insect resistant transgenic cotton in bed planted wheat. Europ J Agron. 2016; 75: 33–41.

[5] TanveerM, Anjum SA, HussainS, CerdàA, AshrafU. Relay cropping as a sustainable approach: problems and opportunities for sustainable crop production. Environ Sci Pollut Res. 2017; 24(8): 6973–6988. doi: 10.1007/s11356-017-8371-4 28083744

[6] SajjadA, AnjumSA, AhmadR, WaraichEA. Relay cropping of wheat (*Triticum aestivum* L.) in cotton (*Gossypium hirsutum* L.) improves the profitability of cotton-wheat cropping system in Punjab, Pakistan. Environ Sci Pollut Res. 2018; 25(1): 782–789. doi: 10.1007/s11356-017-0422-3 29063403

[7] RazzaqA, ZafarMM, AliA, HafeezA, BatoolW, ShiY, et al. Cotton germplasm improvement and progress in Pakistan. J Cotton Res. 2021; 4(1): 1–14.

[8] TariqM, FatimaZ, IqbalP, NaharK, AhmadS, HasanuzzamanM. Sowing dates and cultivars mediated changes in phenology and yield traits of cotton-sunflower cropping system in the arid environment. Int J Plant Prod. 2021; 15(2): 291–302.

[9] MubeenK, AfzalMN, TariqM, AhmadM, MuhammadD, ShehzadM, et al. Sowing date influences cotton leaf curl disease (CLCuD) incidence and productivity of non-Bt cotton cultivars. Pure App Biol. 2022; 11(1): 26–34.

[10] KrzyzanowskiFC, DeloucheEJC. Germination of cotton seed in relation to temperature. Rev Bras Sementes. 2011; 33(3): 543–548.

[11] ReddyKR, BrandD, WijewardanaC, GaoW. Temperature effects on cotton seedling emergence, growth, and development. Agron J. 2017; 109: 1379–1387.

[12] PettigrewWT. Improved yield potential with an early planting cotton production system. Agron J. 2002; 94: 997–1003.

[13] MahmoodT, ArshadM, GillMI, MahmoodHT, TahirM, HussainS. Burewala strain of cotton leaf curl virus: A threat to CLCuV cotton resistance varieties. Asian J Plant Sci. 2003; 2: 968–970.

[14] FarooqA, FarooqJ, MahmoodA, ShakeelA, RehmanKA, BatoolA, et al. An overview of cotton leaf curl virus disease (CLCuD) a serious threat to cotton productivity. Aust J Crop Sci. 2011; 5(13): 1823–1831.

[15] FarooqJ, FarooqA, RiazM, ShahidMR, SaeedF, IqbalMS, et al. Cotton leaf curl virus disease a principle cause of decline in cotton productivity in Pakistan (a mini review). Can J Plant Prot. 2014; 2: 9–16.

[16] MahmoodT, JamilI, TahirM, HussainS. MahmoodHT. Influence of weather variables on Cotton Leaf Curl Disease (CLCuD) in cotton (*Gossypium hirsutum* L.) planted in three districts of the Punjab. Int J Cotton Res Technol. 2014; 56(1–4): 50–59.

[17] TahirM, TariqM, MahmoodHT, HussainS. Effect of sowing dates on incidence of cotton leaf curl virus on different cultivars of cotton. Plant Pathol J. 2004; 3: 61–64.

[18] AliH, HussainGS, HussainS, ShahzadAN, AhmadS, JaveedHMR, SarwarN. Early sowing reduces cotton leaf curl virus occurrence and improves cotton productivity. Cerc Agron Mold. 2014; 47: 71–81.

[19] TariqM, AfzalMN, MuhammadD, AhmadS, ShahzadAN, KiranA, et al. Relationship of tissue potassium content with yield and fiber quality components of Bt cotton as influenced by potassium application methods. Field Crops Res. 2018; 229: 37–43.

[20] JabranK, NawazA, UludagA, AhmadS, HussainM. Cotton relay intercropping under continuous cotton-wheat cropping system. Cotton Production and Uses, 2020: 311.

[21] WangG, FengL, LiuL, ZhangY, LiA, WangZ, et al. Early relay intercropping of short-season cotton increases lint yield and earliness by improving the yield components and boll distribution under wheat-cotton double cropping. Agriculture. 2021; 11: 1294. doi: 10.3390/agriculture11121294

[22] MahmoodA, AnjumFH, AliA. Rice planting geometry facilitating relay cropping at zero tillage. Int J Agr Bio. 2003; 5: 435–437.

[23] KumarS, BahlJR, BansalRP, GuptaAK, SinghV, SharmaS. High economic returns from companion and relay cropping of bread wheat and menthol mint in the winter–summer season in north Indian plains. Ind Crops Products. 2002; 15: 103–114.

[24] DuaVK, GovindakrishnanPM, LalSS. Evaluation of wheat-potato relay intercropping system in the mid hills of Shimla. Ind J Agric Res. 2007; 41: 142–147.

[25] BitewY, AsargewF. Rice (Oryza sativa L.) and chickpea (*Cicer aritinum* L) relay intercropping systems in an additive series experiment in rain fed lowland ecosystem of fogera vertisols. Sci. J Review, 2015; 4: 10–16.

[26] GaudinACM, JanovicekK, MartinRC, DeenW. Approaches to optimizing nitrogen fertilization in a winter wheat-red clover (*Trifolium pratense* L.) relay cropping system. Field Crops Res. 2014; 155: 192–201.

[27] YirzaglaJ, DenwarNN, DogbeW, KantonRAL, InusahIYB, AkakpoDB, et al. Compatibility of millet and legume under relay cropping condition. J Biol Agric Health. 2013; 3: 86–91.

[28] PunyalueaA, JongjaideeJ, JamjodS, RerkasemB. Reduce burning in maize production by relay cropping with legume. Agric Agric Sci Procedia. 2015; 5: 17–21.

[29] IslamMR, UddinMK, AliMO. Performance of lentil varieties under relay and minimum tillage conditions in T. Aman rice. Bangladesh J Agric Res. 2015; 40: 271–278.

[30] YuJ, BoydNS. Relay-cropping and fallow programs for strawberry-based production system: Effects on crop productivity and weed control. Hortsci. 2018; 53(4): 445–450.

[31] SinghM, SidhuHS, MahalJS, ManesGS, JatML, MahalAK, et al. Relay sowing of wheat in the cotton–wheat cropping system in North-West India: technical and economic aspects. Exp Agric. 2017; 53(4): 539–552.

[32] ZhangL, Van der WerfW, ZhangS, LiB, SpiertzJHJ. Growth, yield and quality of wheat and cotton in relay strip intercropping systems. Field Crops Res. 2007; 103: 178–188.

[33] ZhangL, Van der WerfW, BastiaansL, ZhangS, LiB, SpiertzJHJ. Light interception and utilization in relay intercrops of wheat and cotton. Field Crops Res. 2008; 107: 29–42.

[34] ShahMA, HussainM, NawazA, JabranK, FarooqS, FarooqM. Relay intercropping improves growth and fiber quality of Bt cotton. Intl J Agric Biol. 2019; 22: 1539–1546.

[35] KamrozzamanMM, KhanMAH, AhmedS, QuddusAR. On-farm evaluation of production potential and economics of Wheat-Jute-T. aman rice-based cropping system. J Bangladesh Agric Uni. 2015; 13(1): 93–100.

[36] TomerSS, TiwariAS. Production potential and economics of different crop sequences. Indian J Agron. 1990; 35 (1&2): 30–35.

[37] MukherjeeD. Evaluation of different crop sequence production potential, economics and nutrient balance under new alluvial situation of NEPZ. Int J Hort Agric. 2016; 1(1): 5. doi: 10.15226/2572-3154/1/1/00102

[38] SteelRGD, TorrieJH, DickeyDA. Principles and Procedures of Statistics: abiometrical approach. 3rd Ed. McGraw Hill, Inc.Book Co. New York (U.S.A.). 1997; 352–358.

[39] KhanMB, KhanM, HussainM, FarooqM, JabranK, LeeDJ. Bio-economic assessment of different wheat-canola intercropping systems. Int J Agric Biol. 2012; 14: 769–774.

[40] GouF, van IttersumMK, WangG, van der PuttenPEL, van der WerfW. Yield and yield components of wheat and maize in wheat–maize intercropping in the Netherlands. Europ J Agron. 2016; 76: 17–27.

[41] El-HawaryNA. Formulas for relay intercropping and crop sequences systems evaluation, J App Sci Res. 2009; 5 (21): 2074–2082.

[42] ZaherSh R Abd EL, AliAM. Relay intercropping of cotton with wheat under different nitrogen fertilizer levels. Egypt J Agron. 2012; 34(2): 283–299.

[43] ShahMA, ManafA, HussainM, FarooqS, Zafar-ul-HyeM. Sulphur fertilization improves the sesame productivity and economic returns under rainfed conditions. Int J Agric Biol. 2013; 15, 1301–1306.

[44] FarooqS, HussainM, JabranK, HassanW, RizwanMS, YasirTA. Osmopriming with CaCl2 improves wheat (*Triticum aestivum* L.) production under water-limited environments. Environmental Science and Pollution Research. 2017; 24(15), 13638–13649. doi: 10.1007/s11356-017-8957-x 28391467

[45] ShahzadM, HussainM, FarooqM, FarooqS, JabranK, NawazA. Economic assessment of conventional and conservation tillage practices in different wheat-based cropping systems of Punjab, Pakistan. Environmental Science and Pollution Research. 2017; 24(31), 24634–24643. doi: 10.1007/s11356-017-0136-6 28913583

